The article "Efficiency of Nanohydroxyapatite on Repairing Type II Diabetes Dental Implant-Bone Defect" was retracted in 2024. Reasons: signs of a paper mill; suspected computer-generated content; unreliable results or conclusions; concerns about the data.

# Efficiency of Nanohydroxyapatite on Repairing Type II Diabetes Dental Implant-Bone Defect

**DOI:** 10.1155/2022/7459139

**Published:** 2022-06-28

**Authors:** Dong Ji, Dapeng Lu

**Affiliations:** ^1^Department of Oral and Maxillofacial Surgery, Shanxi Medical University, Taiyuan, 030001 Shanxi, China; ^2^Capital Medical University, Beijing 10000, China

## Abstract

The purpose of this study was to see how a nanohydroxyapatite (n-HA) composite polyamide 66 (PA66) affected the repair of bone defects in diabetics with titanium implants, as well as to develop experimental materials for the creation of the interface between bone tissue and titanium implants. Rabbit bone marrow mesenchymal stem cells (MSCs) were isolated using n-HA/PA66 composite material, and the effect of coculture with the material on cell proliferation was analyzed after induction of mineralization. Bone defect models of diabetic experimental rabbits and titanium implants were prepared. Normal rabbits with bone defects were used as control (NC group, *N* = 8). After the diabetic bone defect (DM group, *N* = 8) and the implantation of n-HA/PA66 composite material (n-HA/PA66 group, *N* = 8), the differences in body weight, blood glucose, scanning electron microscopy of the implant-bone interface, bone mineral density, new bone trabecular parameters, histomorphology, and biomechanical properties of the implant-bone interface were compared and analyzed. In vitro test results showed that MSC cell growth could be promoted by mineralization induction, the cell growth condition was good after coculture with n-HA/PA66, and the proliferation activity of MSCs was not affected by the material. In vivo test results showed that the body weight of the DM group and n-HA/PA66 group was considerably inferior to that of the NC group, and the blood glucose was dramatically superior to that of the NC group (*P* < 0.05). However, the body weight of the n-HA/PA66 group was dramatically superior to that of the DM group (*P* < 0.05). The bone mineral density, bone volume fraction (BV/TV), bone surface area fraction (BS/BV), bone trabecular thickness (Tb.Th), bone trabecular number (Tb.N), bone trabecular area, and biomechanical properties in the DM group were considerably inferior to those in the NC group and n-HA/PA66 group (*P* < 0.05). The trabecular space (Tb.Sp) in the NC group and n-HA/PA66 group was dramatically superior to that in the NC group (*P* < 0.05). The bone mineral density, BV/TV, BS/BV, Tb.Th, Tb.N, trabecular area, and biomechanical properties of the n-HA/PA66 group were dramatically superior to those of the NC group (*P* < 0.05), while Tb.Sp was considerably inferior to that of the NC group (*P* < 0.05). These findings showed that the n-HA/PA66 material had good biocompatibility and minimal cytotoxicity, and that filling the space between the surrounding bone and the titanium implant can enhance bone repair. This research paved the way for future research into the tissue-engineered bone in the field of oral surgery.

## 1. Introduction

Dental implant surgery is currently one of the main surgical methods for the treatment of dentition defects in clinical practice, which has the advantages of short time, high safety, and small trauma [1]. Dental implant surgery is often used for adults with fully developed teeth and bones, and there will be no obvious inflammation or damage to the soft tissues in the oral cavity after surgery [2]. With the gradual improvement of people's living standards, the incidence of diabetes also presents an increasing trend year by year [3]. At present, diabetes has become a chronic noncommunicable disease with the highest incidence, which seriously harms people's physical and mental health [4]. Type II diabetes affects more than 90% of diabetics, with clinical symptoms such as hyperglycemia, insulin insufficiency, and insulin resistance, all of which raise the risk of consequences like cardiovascular disease, stroke, and kidney failure [5, 6]. Some studies suggested that type I diabetes can lead to decreased bone mass, but the effect of type II diabetes has not been proven yet [7]. Patients with type II diabetes have a significantly higher risk of fracture, and all clinical consensus is that diabetes can affect the formation of new bone, bone ultrastructure, and bone quality of patients [8]. Because of the hyperglycemic milieu in the patient's body and pathological changes in some microvessels, the proliferation and differentiation of osteogenic extractions can be impeded to some extent after dental implant surgery for individuals with type II diabetes. It may also promote osteoclast differentiation, which in turn affects the bone-binding effect of implants. Therefore, dental implant surgery for patients with type II diabetes has certain safety risks [2, 9]. Studies confirmed that the environment of high blood sugar in the body of diabetes patients can aggravate the inflammatory response and cause the dysfunction of the immune system [10]. As a result, dental implant repair for diabetic patients may have an impact on the repair effect, and patient bone defect healing after treatment has become one of the most pressing issues to be solved in clinical surgery.

Immediate implant materials that can be used to guide bone tissue growth and repair have been sought to improve the success rate of implants and reduce patients' posttreatment evaluation due to infection, malignancy, or periodontal disease. Recent studies suggested that the autologous jaw has good biocompatibility, bone conduction, bone induction, and high safety advantages in immediate implantation, but certain complications may be induced when the autologous jaw is used for bone extraction [11, 12]. Patients who have allogeneic bone transplants, on the other hand, are more likely to develop a rejection reaction and infection [13]. The structure of nanohydroxyapatite (n-HA) is very similar to the crystal structure of the inorganic component of human bone, and it has good biological activity, no cytotoxicity, no immunogenicity, and good degradation performance [14]. Studies confirmed that n-HA can be replaced by newborn bone tissue in a short time and can induce and stimulate the proliferation and differentiation of local osteocytes [15]. However, a single material cannot well meet the clinical needs, and pure n-HA has high brittleness and low strength [16]. Therefore, the emergence and development of composite materials provide a new idea for biomedical materials of human tissues.

To explore the effect of type II diabetes mellitus on the healing of implant-bone defects and the promoting healing effect of n-HA/polyamide 66 (PA66) filling composite artificial bone material, n-HA/PA66 composite porous artificial bone was prepared by using n-HA and PA66 materials firstly. After being isolated, the proliferative activity of rabbit bone marrow mesenchymal stem cells (MSCs) was assessed, as well as the MSCs' biocompatibility and cytotoxicity after coculture with n-HA/PA66. Secondly, the diabetic and implant-bone defect models were constructed, and the changes in body weight and blood glucose levels in each group were analyzed. Finally, n-HA/PA66 material was filled in the implant-peripheral bone space to analyze its effects on bone density, histomorphology, new bone trabeculae, and biomechanics at the bone healing site. This study is aimed at providing an experimental basis for improving the therapeutic effect of dental implant surgery in patients with type II diabetes.

The rest of the paper is organized as follows: Section 2 gives materials and methods, Section 3 gives results, Section 4 gives discussion, and the conclusion is mentioned in Section 4.

## 2. Materials and Methods

In this section, we will discuss the isolation and culture of rabbit bone marrow mesenchymal stem cells (MSCs), preparation and characterization of n-HA/PA66 biomimetic bone, MSC proliferation detected by methyl tetrazolium (MTT) assay, osteogenic ability of bmscs detected by alkaline phosphatase (ALP), preparation and grouping of animal models, bone defect specimens observed by scanning electron microscopy, radiographic examination of bone defect specimens, histological observation of bone defect specimens, biomechanical determination of bone defect specimens, and statistical treatment in detail.

### 2.1. Isolation and Culture of Rabbit Bone Marrow Mesenchymal Stem Cells (MSCs)

The head of the test subject was tapped, and the tibia was taken under aseptic conditions and soaked in 75% alcohol and D'hanks reagent for 20 s and 10 min, respectively. The fat layer was removed from the bone marrow, and the cells were suspended in low-glucose Dulbecco's modified Eagle medium (DMEM). Cells were stratified with 5 mL Percoll separation solution, and the cell suspension was prepared after centrifugation. The cells were inoculated in the culture dish with DMEM containing 10% fetal bovine serum and 1% penicillin plus streptomycin. The cells were cultured in a 5% CO_2_ incubator at 37°C, and the fluid was changed once for 3 days. When the confluence of cells reached 90%, the cells were subcultured.

### 2.2. Preparation and Characterization of n-HA/PA66 Biomimetic Bone

PA66 powder was dissolved in alcohol solution, and n-HA slurry was prepared by wet synthesis with hydrothermal treatment. n-HA slurry was slowly added to the PA66 reagent with a mass ratio of 3 : 1 and stirred continuously for 2 h under the constant humidity condition of 55%, to obtain the n-HA/PA66 composite solution. n-HA/PA66 composite solution was poured into the mold, and porous n-HA/PA66 composite artificial bone material was prepared by the phase transfer method.

### 2.3. MSC Proliferation Detected by Methyl Tetrazolium (MTT) Assay

Cut to size, the porous n-HA/PA66 composite artificial bone material was inserted at the bottom of a 96-well plate. For one day, the material was soaked in a mineralized induction solution. MSCs after mineralized induction for 7 days were inoculated into the well plate at a density of 1 × 10^6^. Samples were taken at 0.5 d, 1 d, 3 d, and 7 d after routine culture, and cell count was performed after trypsin digestion. MTT colorimetric test was performed, and 20 *μ*L MTT reagent was added to the cell wells and incubated in the cell incubator for 4 h. Then, a 150 *μ*L dimethyl sulfoxide (DMSO) reagent was added and gently shaken for 10 min. The absorbance value of each well was measured at 570 nm by a multifunction microplate analyzer, and the cell growth curve was plotted.

### 2.4. Osteogenic Ability of BMSCs Detected by Alkaline Phosphatase (ALP)

The cells were cocultured according to the above method, and ALP activity was detected using an ALP kit at 0.5 d, 1 d, 3 d, and 7 d of mineralization induction and culture, respectively. Cells in each group were tested three times, and the ALP level of cells was compared with the mean value.

### 2.5. Preparation and Grouping of Animal Models

With eight rabbits in each group, twenty-four New Zealand white rabbits were randomly assigned to the normal control group (NC), diabetes model group (DM), and n-HA/PA66 stent implantation group (n-HA/PA66) in terms of treatment approaches.

After the subjects were weighted, the skin was prepared and disinfected in the ear margin vein, and the animals were anesthetized by intravenous injection of 40 mg/kg 3% pentobarbital sodium solution. 50 mg/mL and 100 mg/mL alloxan were injected slowly into the ear vein, and 10 mL 5% glucose was injected subcutaneously 2 h, 4 h, and 6 h after injection to prevent hypoglycemia in animals. They were reared in separate cages and given drinking water containing 10% glucose for 1 day. Blood glucose was detected every 24 hours. When the blood glucose of model animals reached stable, blood glucose was detected every three days. When the animal's blood glucose (fibrinogen) level exceeded 19.4 mmol/L, 2.5 U/kg of insulin was injected subcutaneously. After modeling, blood glucose was tested every seven days. When the fibrinogen level was always higher than 13.9 mmol/L, the diabetes model was considered as successful.

At the upper end of the subject's lateral femur, the skin and subcutaneous tissue were sliced along the long axis, and the muscle layer was separated to expose the greater trochanter region of the femur. The periosteum was removed, and an implant socket with a diameter of 2 mm and a depth of 7 mm was made. The implants were inserted at 2 cm after being washed and cooled in isotonic saline, and bone defects of 2 mm, 3 mm, and 2 mm were obtained from the central side. After the wound area was flushed with normal saline, the bleeding was stopped and disinfected. Animals in the NC group and DC group were not implanted with any material, while those in the n-HA/PA66 group were implanted with MSCs/n-HA/PA66 material. Three days following the operation, stratified sutures, cage feeding, and continuous injection of gentamicin 80,000 U/d were used.

### 2.6. Bone Defect Specimens Observed by Scanning Electron Microscopy

Femur samples of each group were collected at 8 w after surgery. After being rinsed with normal saline, the tissue was fixed with a 2% glutaraldehyde solution, and then, the samples were observed and recorded under a scanning electron microscope.

### 2.7. Radiographic Examination of Bone Defect Specimens

X-ray images were utilized to scan bone specimens. The scanning parameters were set as the voltage of 45 kV, current of 100 mA, and scanning time of 0.12 s. Bone mineral density (BMD) was analyzed at the implant-bone tissue interface using automatic image analysis software, and the sampling area was 1.0 mm × 1.5 mm.

*μ*CT images were utilized to scan bone specimens. The scanning parameters were set as the voltage of 80 kV, current of 50 mA, and resolution of 14.95 *μ*m. Image processing software was employed for the 3D reconstruction of the image, and regions of interest were marked. Regarding the Standard of Hounsfield units, the new bone tissue at the bone defect site was analyzed. The analysis parameters included bone volume fraction (BV/TV), bone surface area fraction (BS/BV), bone trabecular thickness (Tb.Th), bone trabecular number (Tb.N), and bone trabecular space (Tb.Sp).

### 2.8. Histological Observation of Bone Defect Specimens

Bone samples were collected from each group, and the tissues were fixed with 10% neutral formalin for 1 d. After the tissues were cleaned with phosphoric acid buffer, the tissues were decalcified with 10% EDTA decalcification solution for 2 w. The tissues were dehydrated with 70 percent, 80 percent, 90 percent, 95 percent, 95 percent, 95 percent, and 100 percent ethanol solutions and then transparently treated with xylene solution and embedded in paraffin solution. Using a slicer, the paraffin tissue was sectioned into 5 *μ*m paraffin sections and dried at 45°C. Then, the tissues were rehydrated with 95%, 95%, 80%, and 75% ethanol solutions and rinsed with distilled water. The tissue was stained with hematoxylin solution first and then dyed with eosin solution after water flushing. After water flushing, the tissue was dehydrated and treated transparently and finally sealed with a neutral gum solution. The histomorphological changes of specimens were observed and recorded under a microscope.

### 2.9. Biomechanical Determination of Bone Defect Specimens

Femur samples were collected at 14 d, 30 d, 60 d, and 90 d after surgery, and bone specimens were separated along the original incision. The tissues were fixed with 10% formaldehyde solution, and the biomechanical properties of the samples were measured with a universal mechanical testing machine at a loading speed of 2 mm/min.

### 2.10. Statistical Treatment

All experimental data were organized and analyzed using SPSS 19.0 and were expressed by mean ± standard deviation (*x̅*±*s*). The differences between groups were statistically analyzed using a one-way analysis of variance (ANOVA), and *P* < 0.05 was considered statistically significant.

## 3. Results

In this section, we will discuss the osteogenesis evaluation of rabbit MSCs cocultured with n-HA/PA66, changes in body weight and blood glucose after n-HA/PA66 repair, scanning electron microscope observation of bone tissue after n-HA/PA66 repair, radiographic examination of bone tissue after n-HA/PA66 repair, morphological observation of bone tissue after n-HA/PA66 repair, and a biomechanical test of bone tissue after n-HA/PA66 repair in detail.

### 3.1. Observation of Rabbit MSCs

The isolated rabbit MSCs were cultivated in primary culture, and the cultured cells' growth morphology was examined under an inverted microscope. The results revealed that cells in normal culture were tightly packed, with the majority of cells resembling a spindle shape and a few triangular or star-shaped cells. The proliferation rate of cells grew rapidly after mineralization-induced culture, and the number of cells and slender axons joined, grouped, and merged, resulting in a clumped growth condition overall. The rabbit MSCs' growth status was examined as shown in Figure 1.

### 3.2. Cell Adhesion after Coculture of n-HA/PA66 with Rabbit MSCs

Scanning electron microscopy was employed to evaluate the adhesion of n-HA/PA66 composite artificial bone material and rabbit MSCs after coculture (Figure 2). n-HA/PA66 composite artificial bone material had a porous structure, which was conducive to the growth of cells inward. After coculture of n-HA/PA66 composite artificial bone material with rabbit MSCs, the cells were attached to the surface of the material. Furthermore, the cell development morphology was rather diversified, with cells growing inward along the pore surface and connecting into slices.

### 3.3. Cell Proliferation Evaluation after Coculture of n-HA/PA66 with Rabbit MSCs

MTT assay was adopted to evaluate the difference in proliferation activity of MSCs after normal culture (Nor), mineralization induction (MI), and n-HA/PA66 coculture (coculture).  Figure 3 shows that as culture time went on, the proliferation activity of cells in the Nor, MI, and coculture groups increased gradually, with the Nor group always having the highest proliferation activity. The proliferative activity of the three groups did not differ significantly after comparison (*P* > 0.05).

### 3.4. Osteogenesis Evaluation of Rabbit MSCs Cocultured with n-HA/PA66

The difference in the osteogenic ability of MSCs after normal culture (Nor), mineralization induction (MI), and n-HA/PA66 coculture (coculture) was evaluated by the ALP activity test (Figure 4). Alkaline phosphatase activity of MSCs in the MI group and coculture group was always considerably increased than the Nor group after 12 h of culture (*P* < 0.05). There was no significant difference in ALP activity of MSCs between the MI group and the coculture group at different time points (*P* > 0.05).

### 3.5. Changes in Body Weight and Blood Glucose after n-HA/PA66 Repair

In Figure 5, the effect of diabetes modeling was tested by detecting and recording changes in body weight and blood glucose levels of experimental rabbits in the three groups. Experimental rabbits in the NC group had lower body weight and blood glucose levels. The experimental rabbits in the NC group had relatively steady body weight and blood glucose levels. The weight of experimental rabbits in the DM and n-HA/PA66 groups declined at first and then grew, and blood glucose levels steadily increased and tended to remain steady. The body weight of the DM group and n-HA/PA66 group was always obviously inferior to that of the NC group after seven days of modeling (*P* < 0.05). After one day of modeling, the blood glucose level of the DM group and n-HA/PA66 group was always evidently superior (*P* < 0.05). The weight of experimental rabbits in the n-HA/PA66 group was always substantially higher than the DM group after seven days of modeling (*P* < 0.05).

### 3.6. Scanning Electron Microscope Observation of Bone Tissue after n-HA/PA66 Repair

A scanning electron microscope was employed to observe the structural changes of the three groups after repair (Figure 6). In the NC group, only a small amount of bone union occurred, while in the DM group, the state of the bone union was worse. In the n-HA/PA66 group, the implant was tightly bound to the new bone with less space.

### 3.7. Radiographic Examination of Bone Tissue after n-HA/PA66 Repair

At 14 days, 30 days, 60 days, and 90 days after therapy, X-ray imaging equipment was used to assess changes in bone mineral density in the three groups (Figure 7). With the extension of implantation time, the bone mineral density of experimental rabbits in each group showed a trend of gradual increase. Only bone mineral density in the DM group was remarkably decreased 30 d after implantation (*P* < 0.05), and bone mineral density in the n-HA/PA66 group was notably increased 60 d after implantation (*P* < 0.05). In addition, bone mineral density in the n-HA/PA66 group was notably increased 30 days after implantation relative to the DM group (*P* < 0.05).

*μ*CT imaging was performed to evaluate the changes of trabecular parameters of new bone at the site of bone injury in the three groups at 90 d after treatment (Figure 8). BV/TV, BS/BV, Tb.Th, and Tb.N of trabecular bone of experimental rabbits in the DM group were remarkably decreased than in the NC group (*P* < 0.05), while the levels of Tb.Sp were on the opposite. BV/TV, BS/BV, TB.Th, and Tb.N in only the n-HA/PA66 group were notably increased (*P* < 0.05), while the levels of Tb.Sp were remarkably decreased (*P* < 0.05).

### 3.8. Morphological Observation of Bone Tissue after n-HA/PA66 Repair

HE staining sections of bone tissue were made, and histomorphological changes were observed (Figure 9).  Figure 9(a) shows that 90 days after surgery, the edge of the bone defect in experimental rabbits in the NC and DM groups was apparent, and only a tiny quantity of new tissue was formed, whereas a substantial amount of connective tissue emerged at the defect site. The number of osteoblasts and new tissue at the site of the bone defect was considerably lower in the DM group than in the NC group. Nanomaterials, callus, osteoid, and new capillaries were identified at the bone defect interface in the n-HA/PA66 group compared to the NC and DM groups.

The percentage area of bone trabecular bone at 14, 30, 60, and 90 d after the operation was determined. In Figure 9(b), with the extension of postoperative time, the trabecular area of experimental rabbits in the three groups gradually increased. The bone trabecular area in the DM group was remarkably decreased 30 days after surgery versus the NC group (*P* < 0.05). The trabecular area of the n-HA/PA66 group increased greatly 14 days after surgery (*P* < 0.05). The trabecular area of the n-HA/PA66 group was notably increased 14 days after surgery relative to the DM group (*P* < 0.05).

### 3.9. Biomechanical Test of Bone Tissue after n-HA/PA66 Repair

The differences in the biomechanical properties of bone tissues were detected and evaluated, and the results are shown in Figure 10. The biomechanical properties of bone tissue in the NC group, DM group, and n-HA/PA66 group showed a trend of gradual increase with the increase of treatment time. Compared with the NC group, the biomechanical properties of bone tissue in the DM group were remarkably decreased 30 days after surgery (*P* < 0.05), while the biomechanical properties of bone tissue in the n-HA/PA66 group were notably increased (*P* < 0.05). The biomechanical properties of bone tissue in the n-HA/PA66 group were notably increased relative to the DM group (*P* < 0.05).

## 4. Discussion

The problem of dental diseases is growing increasingly prevalent as people's living standards and quality of life increase. For individuals who have lost teeth, implant repair can restore dental tissue to a state that is extremely comparable to natural teeth [17]. Dental implant restoration technology mainly uses artificial materials to synthesize implants similar to the structure of natural tooth roots. The implant is then surgically implanted into the alveolar bone of the patient. The prosthesis is attached to the implant, which is closely integrated with the alveolar bone. This technique allows the implant to operate similarly to a natural tooth [18]. Massive studies confirmed that the stability of dental implants in patients with type II diabetes after dental implant surgery is worse than that in normal people [19, 20]. This may be due to the high level of blood glucose in diabetic patients, which may cause inflammation to a certain extent and reduce the healing ability and immune function of tissues, thus weakening the bone-binding ability of implants [21]. Therefore, to improve the bone-binding effect of diabetic implants, filling material for the implant-peripheral bone interface was fabricated, and its effect on bone healing effect was analyzed.

At present, the most common polymer composite materials include hydroxyapatite (HA), polyamide, and polylactic acid, among which HA has good biocompatibility. Nevertheless, its strength is low and brittleness is high, so its damage resistance is not high in the actual physiological environment [22]. To meet the needs of bone scaffold materials, porous artificial bone materials with nanometer HA and PA66 were prepared. The pore size of n-HA/PA66 porous composite artificial bone material was 300 *μ*m, and there were abundant micropore structures in the material matrix connected [23]. The amount of solvent, the rate of heating, and the temperature control time can all affect porosity. However, the apatite concentration of n-HA/PA66 at the nanoscale level was similar to that of normal bone, laying the groundwork for the biological activity of the compound. Good bone tissue engineering materials, good biocompatibility, and physical compatibility are the basic requirements of composite scaffold materials, which provide a site for cell growth, differentiation, and proliferation [24, 25]. In this research, the prepared n-HA/PA66 material was cocultured with MSCs. By observing the cell growth status and proliferation activity, it was found that MSCs could grow into the pores of n-HA/PA66 material, and there was no significant difference in proliferation activity between MSCs cultured under conventional conditions. It was also found that ALP staining was positive for MSCs after coculture, indicating that n-HA/PA66 material had good biocompatibility and no cytotoxicity and could not affect the osteogenic differentiation of MSCs.

Diabetes can affect blood transport in the body, reduce the distribution of blood vessels in bone tissue, and increase the permeability of microcirculation capillaries. In turn, it affects the matrix composition and content around blood vessels and ultimately leads to delayed or nonunion of bone healing and even ischemic necrosis of bone in severe cases [26]. This work was to understand the effect of n-HA/PA66 material prepared in this experiment on bone defect healing of diabetic implants. Alloxan can selectively destroy pancreatic *β* cells, cause cell failure, block cell secretion of insulin, and then cause diabetes [27]. The results showed that the weight of experimental rabbits was considerably inferior to that of normal rabbits, while the blood glucose level was always higher than that of normal rabbits. These results indicated that the diabetic rabbit animal model was successfully prepared. After the implant-bone defect model was prepared, radiographic and histomorphological observations showed that the defect parts were completely repaired, indicating that the implant-bone defect animal model was successfully constructed, which laid a foundation for subsequent research. Insulin has a vital function in the regeneration and repair of bone tissue [28]. The experimental rabbits with diabetes had a considerably lower bone density, trabecular area of new bone, and biomechanical qualities than those with typical bone defects, and less new tissue and blood vessels grew in the bone defects. These findings suggested that diabetes can interfere with the process of tissue repair and regeneration in rabbits with bone abnormalities, lowering the tissue's biological strength.

Subsequently, the effect of n-HA/PA66 porous composite artificial bone material on the bone binding ability of diabetic rabbits with the implant-bone defect was compared and analyzed. The results showed that after n-HA/PA66 supplementation, the bone mineral density, BV/TV, BS/BV, Tb.Th, and Tb.N levels, trabecular area, and biomechanical properties of rabbits were significantly increased, whereas the Tb.Sp level was significantly decreased when compared to the normal implant-bone defect rabbit model and the diabetic implant-bone defect rabbit model. The results showed that n-HA/PA66 could promote the healing of bone defects in diabetic animals. This was because n-HA/PA66 composite material with MSCs had a structure similar to the natural bone interface, and the porous structure provided a site for the growth, proliferation, and differentiation of osteoblasts and promoted the osteogenesis of MSCs [29, 30]. The aforesaid findings revealed that the MSC composite n-HA/PA66 material developed had strong bone compatibility, biodegradability, and bone conductivity, as well as being conducive to the formation of blood vessels and cells, laying a solid basis for new bone and implant-bone binding.

## 5. Conclusion and Future Work

In this research, nanoscale n-HA/PA66 porous artificial bone material was prepared to promote the osseous binding between implants and surrounding bone tissue. After coculture with MSCs, it was found that the material had good biocompatibility, no cytotoxicity, and did not affect the proliferation and osteogenic differentiation of MSCs. Following that, the diabetes implant-bone defect animal model was produced and filled with MSC composite and n-HA/PA66 material at the same time. The substance was discovered to promote osseous adhesion between the implant and the surrounding bone tissue, and it might be used to correct implant-bone defects. However, only animal models were used to examine the material's ability to heal bone abnormalities caused by diabetes implants, and the material's efficacy and safety will be confirmed in clinical trials in the future. In conclusion, this study can provide an experimental basis for the promotion and application of oral implant surgery and the improvement of periodontal disease in patients with type II diabetes.

## Figures and Tables

**Figure 1:** Microscopic observation of primary rabbit MSC culture and mineralized induction culture (×100).

**Figure 2:** Scanning electron microscope observation of n-HA/PA66 cocultured with rabbit MSCs.

**Figure 3:** MTT assay of proliferation activity of rabbit MSCs.

**Figure 4:** Alkaline phosphatase activity of rabbit MSCs. (a) Observed by ALP staining; (b) ALP activity detection results; compared with the Nor group, ^∗^*P* < 0.05.

**Figure 5:** Effects of n-HA/PA66 implantation on body weight and blood glucose level of experimental rabbits. (a) The change in body weight; (b) the change of blood glucose level; compared with the NC group, ^∗^*P* < 0.05; compared with the DM group, ^#^*P* < 0.05.

**Figure 6:** Scanning electron microscope observation of the effect of n-HA/PA66 implantation on bone trauma in experimental rabbits (×25,000; ×10,000).

**Figure 7:** Effect of n-HA/PA66 implantation on the bone mineral density of the new bone in experimental rabbits. Compared with the NC group, ^∗^*P* < 0.05; compared with the DM group, ^#^*P* < 0.05.

**Figure 8:** Effects of n-HA/PA66 implantation on trabecular parameters of new bone in experimental rabbits. (a) BV/TV; (b) BS/BV; (c) Tb.Th; (d) Tb.N; (e) Tb.Sp; compared with the NC group, ^∗^*P* < 0.05; compared with the DM group, ^#^*P* < 0.05.

**Figure 9:** Bone histomorphological evaluation of n-HA/PA66 implantation in experimental rabbits. (a) Morphological observation after HE staining (×40); (b) the percentage of the bone trabecular area; compared with the NC group, ^∗^*P* < 0.05; compared with the DM group, ^#^*P* < 0.05.

**Figure 10:** Biomechanical evaluation of n-HA/PA66 implantation on experimental rabbit bone tissue. Compared with the NC group, ^∗^*P* < 0.05; compared with the DM group, ^#^*P* < 0.05.

## Data Availability

The data that support the finding of this study are available from the corresponding upon reasonable request.
